# Identification of Navel Orange Diseases and Pests Based on the Fusion of DenseNet and Self-Attention Mechanism

**DOI:** 10.1155/2021/5436729

**Published:** 2021-09-02

**Authors:** Yin'e Zhang, Yong Ping Liu

**Affiliations:** School of Mathematics and Computer Science, Gannan Normal University, Ganzhou, Jiangxi 341000, China

## Abstract

The prevention and control of navel orange pests and diseases is an important measure to ensure the yield of navel oranges. Aiming at the problems of slow speed, strong subjectivity, high requirements for professional knowledge required, and high identification costs in the identification methods of navel orange pests and diseases, this paper proposes a method based on DenseNet and attention. The power mechanism fusion (DCPSNET) identification method of navel orange diseases and pests improves the traditional deep dense network DenseNet model to realize accurate and efficient identification of navel orange diseases and pests. Due to the difficulty in collecting data of navel orange pests and diseases, this article uses image enhancement technology to expand. The experimental results show that, in the case of small samples, compared with the traditional model, the DCPSNET model can accurately identify different types of navel orange diseases and pests images and the accuracy of identifying six types of navel orange diseases and pests on the test set is as high as 96.90%. The method proposed in this paper has high recognition accuracy, realizes the intelligent recognition of navel orange diseases and pests, and also provides a way for high-precision recognition of small sample data sets.

## 1. Introduction

The output of navel oranges in China ranks among the top in the world, but, due to the impact of navel orange diseases and pests, the output and quality of navel oranges have declined to varying degrees. Diseases and pests of navel oranges can be detected visually, because they often affect the shape or color of fruits, leaves, stems, and other parts of the plant [1]. Farmers must detect the diseased parts and conditions as early as possible before the navel orange disease spreads in the plantation. The traditional method is that farmers rely on human experts to carry out reconnaissance of the plantation in order to find the infected fruit and identify the type of disease. Reconnaissance of the entire plantation is a time-consuming task. In addition, farmers must also pay for experts, and experts are not always available at all times. Due to these problems, researchers have been committed to the application of artificial intelligence methods to the disease detection of navel oranges, and the use of convolutional neural network (CNN) models [2] to identify pests and diseases has become a new trend in the agricultural field.

In recent years, automatic image recognition technology has shown excellent performance in the recognition and classification of plant diseases. There are many ways to identify plant diseases and pests images. Senthilkumar and Kumarasan [3] proposed preprocessing based on bilateral filtering, optimal weighted segmentation (OWS), feature extraction based on Hough Transform (HT), and rough fuzzy artificial neural network (RFANN) based on navel orange. The four types of disease identification, black spot disease, ulcer disease, green disease, and scab, have the accuracy rates of 96.52%, 95.20%, 97.88%, and 97.20%, respectively. Waheed et al. [4] recommended an optimized dense CNN architecture (DenseNet) to identify and classify maize leaf diseases such as northern leaf blight, common rust, grey leaf spot, and healthy leaves. In the experiment, the accuracy rate reached 98.06%. Karthik et al. [5] used three tomato diseases in the Plant Village data set, leaf mold, early blight, and late blight, and reported an attention mechanism embedded in ResNet to identify tomato leaf diseases and the overall accuracy of the classifier. The rate reached 98%. Malathi and Gopinath [6] applied the migration learning method to the pest data set by fine-tuning the superparameters and layers of ResNet-50 model, and the accuracy of the optimized ResNet-50 model reached 95.012%. Malek et al. [7] developed a pest identification and classification model using convolutional neural network (CNN), and the classification accuracy of the model can reach 90%. Ahmad Loti et al. [8] compared the characteristics of pepper diseases and pests extracted by traditional methods with those extracted by deep learning methods; the method based on deep learning features can capture the details and features of different types of pepper diseases and pests. Zekiwos and Bruck [9] developed a model using deep learning technology, CNN, to improve the detection of cotton leaf diseases and insect pests. The *k*-fold cross validation strategy was used to segment and generalize the CNN model. The accuracy of the model in the classification of cotton leaf diseases and insect pests was 96.4%. Chen et al. [10] proposed a new network architecture, Mobile-DANet, to identify maize diseases, and the model achieved an average accuracy of 98.50% on the open maize data set.

## 2. Related Work

The studies in [11, 12] proposed that some feature maps generated by convolution are useless. In order to reduce the influence of redundant features on classification, Hu et al. [13] and Woo et al. [14] introduced an attention mechanism to suppress unnecessary channels. Their methods are more adaptive than dropout [15] and random depth [16]. However, additional branches in each building block increase the overhead of the network. There are many researches on the attention mechanism, which can be generally divided into channel attention mechanism (CAM) and spatial attention mechanism (SAM) (Woo et al.) [14, 17]. In a Network in Network [18], two continuous 11 convolution layers are used to improve the discriminability of the model for local patches. From another perspective, this structure is also a good highway for refining feature mapping network. The study in [19] first proposed the idea of feature reuse, which alleviated the optimization difficulty of deep network. ResNet [20] generalized it with identity mapping. DenseNet [21] further improves the frequency of skipping connections. DenseNet has better presentation capabilities than ResNet because it can produce higher precision with fewer parameters. DenseNet connects all network layers directly to ensure the maximum information flow. In order to maintain the feedforward characteristics, each layer obtains additional input from all previous layers and transmits its own feature map to all subsequent layers. Due to the dense connection mode between layers, DenseNet achieves good performance in image recognition and classification.

In this paper, a simple and effective image recognition network named DCPSNET for navel orange diseases and pests is proposed. The design principle of the network focuses on improving the utilization rate of model parameters, and the self-attention mechanism module is added on the basis of the original DenseNet network, so that the network can better notice the diseases and pests in the training process.

## 3. Data Acquisition and Preprocessing

### 3.1. Navel Orange Image Acquisition

All the data sets of navel orange diseases and insect pests in this paper came from the southern Jiangxi region of Jiangxi Province and were taken on-site by high pixel mobile phones in different orchards. A total of 1157 pieces of navel orange images were collected, and, according to experts in the field of knowledge, image can be divided into health image and plant diseases and pests image including the Sunguo, Canker, leaf miner, *Botrytis cinerea*, and Anthrax.  Table 1 describes the main characteristics of five kinds of navel orange diseases and pests.  Figure 1 shows examples of typical symptoms of these navel orange pests.

### 3.2. Data Enhancement

The images of diseases and pests of navel oranges are extracted and marked by consulting related literature and data combined with main expert knowledge, and then preprocessing techniques such as filtering are performed on the images. Das et al. [22] mentioned the problem of unbalanced data classification by sharpening, resizing, and filling the edges on the original image to increase the number of images in the class whose data set size is smaller compared to other classes. Secondly, in order to diversify the image, a data enhancement scheme is used to enhance the deep convolutional generation adversarial network (DCGAN) [23], with traditional methods such as random vertical or horizontal flipping, random angle rotation, scale transformation, and color dithering to generate new synthesized images to expand the data set and reduce overfitting during network training.

The data set includes 1157 images of navel orange leaves: 74 images of sun fruit disease, 225 images of canker leaf disease, 238 images of canker fruit, 88 images of gray mold, 283 images of leaf miner disease, and 69 images of anthracnose, as well as 180 healthy leaf images. The data distribution of the navel orange image data set is inconsistent, and the number of images of sun fruit disease, anthracnose, and gray mold is relatively less compared to other categories. Therefore, in order to enrich the image and prevent overfitting, this article uses random angle rotation within the range, image translation within ±10%, flip scale transformation within the range, color jitter within the range, Gaussian noise added to the image, and so forth. Data enhancement technology is used to enrich the data set. Through data enhancement, the number of original image samples has been increased by 17 times, and each category has no less than 1000 samples. The specific relevant data sets are shown in Table 2.

In addition to retaining some images to evaluate the effectiveness of the model, according to the method proposed by Too et al. [24], the navel orange pest data are divided into training set and validation set as 8 : 2, and then all image sizes are converted to 224 × 224 using OpenCV technology and saved in jpg image format.

## 4. Establishment of the Model

Inspired by the performance of attention mechanism, this paper embeds position self-attention mechanism (PSAM) and channel self-attention mechanism (CSAM) modules in the network in a serial way. By learning the relationship between channels and the importance of position points to input features, the classification accuracy and the learning ability of micro lesion features are improved.

Therefore, the overall architecture of the model studied in this paper retains the network structure of DenseNet. A total of four density block modules and three training modules are designed. CSAM module is added to each density block module to retain the structure of transition layer. CSAM and PSAM serial modules are added between density block and transition layer, and this network architecture is named DCPSNET.

### 4.1. DenseNet

DenseNet ensures enough information transmission between layers and improves the transmission efficiency of information and gradient in the network. Each layer can directly obtain the gradient value from the loss function and get the input signal directly, which solves the problem of gradient disappearance and reduces the setting of network parameters. DenseNet connects the input images, and the input of each layer is the connection of the output of all the previous layers, so that the eigenvalues can be reused in the whole network:

(1) $$\begin{array}{c} I_{l}=Y_{l}\left(\left[I_{0},I_{1},\ldots ,I_{l-1}\right]\right), \end{array}$$

where *I*_*l*_ is the characteristic output of layer *L*, which passes through a neural network of layer *L*, and the nonlinear transformation of layer *I* represents the combined operation of BN, ReLU, and 3 × 3 conv three functions, where [], represents the splicing operation. All the output feature mapping from layers *I*_0_ to *I*_*l*−1_ are combined together by the channel. The dense block is shown in Figure 2(a).

In order to use downsampling, DenseNet is divided into four density blocks, and transition layers are set between different density blocks to realize downsampling. The transition layer in this paper consists of BN, ReLU, 1 × 1 Conv, and 2 × 2 average pooling, as shown in Figure 2(b).

### 4.2. Position and Channel Attention Mechanisms

Attention mechanism is a selective mechanism, which can pay attention to the important characteristic information of some diseases and pests in navel orange images, while ignoring other unnecessary information. In this paper, position self-attention mechanism (PSAM) is used to capture the spatial dependence of the feature graph between any two positions, and the features of all positions are aggregated and updated by weighted summation. The weight is determined by the feature similarity of the two corresponding positions. Channel self-attention mechanism (CSAM) is used to capture the channel dependence between any two channel graphs. Finally, each channel graph is updated with the weighted sum of all channel graphs. The overall structure of CPSAM is shown in Figure 3.

As can be seen from Figure 3, this paper combines DANet location attention [17], ECANet channel attention [25], and CBAM serial integration mode of channel attention mechanism [14] and finally proposes our CPSAM attention mechanism, which first uses PSAM to detect the target's position in the feature graph and then uses CSAM to mine the interdependence between channel graphs, and the whole attention mechanism is connected in a string. Firstly, *F* ∈ *R*^*C*×*W*×*H*^, and the feature graph generated in the network is input to PSAM module, and then it is sent to convolution layer to generate two new feature graphs *L* and *M*, {*L*, *M*} ∈ *R*^*C*×*H*×*W*^, and then reshape to *R*^*C*×*N*^, *N*=*H* × *W*. Then, matrix multiplication is performed between *M* and *l* transposes, and the softmax layer is applied to calculate the spatial attention graph *P* ∈ *R*^*N*×*N*^.

(2) $$\begin{array}{c} P_{ji}=\sum_{i=1}^{N}{\left(L_{i}\cdot M_{j}\right)}^{-1}*\;\exp\left(L_{i}\cdot M_{j}\right), \end{array}$$

where *p*_*ji*_ is the influence of position *i* on position *j*. The more similar the feature representation of the two positions, the higher the correlation between them. At the same time, feature *F* is sent into the convolution layer to generate a new feature map *O* ∈ *R*^*C*×*H*×*W*^, which is reshaped as  *R*^*C*×*N*^. Then, matrix multiplication is performed between the transposes of *O* and *P*, and the result is reshaped as *R*^*C*×*H*×*W*^. Finally, we multiply *τ* by the scale parameter and use the characteristic *L* to perform the element summation operation to obtain the final output *V* ∈ *R*^*C*×*H*×*W*^. The specific formula is as follows:

(3) $$\begin{array}{c} V_{j}=F_{j}+\tau \sum_{i=1}^{N}\left(p_{ji}\cdot O_{i}\right), \end{array}$$

where *τ* is initialized to 0 and gradually learns to assign more weights. The resulting feature *V* at each location is the weighted sum of the features at all locations and the original features. Therefore, it has a global context view and selectively aggregates contexts according to the spatial attention graph. Then, the feature map *V* ∈ *R*^*C*×*H*×*W*^ generated by PSAM module is used as the input of CSAM feature map, and GAP operation is performed first. The mathematical formula is as follows:

(4) Ζω1,ω2V=ω2ReLUω1V,

where Ζ_{*ω*_1_, *ω*_2_}_(*V*) represents the corresponding relationship between weights *ω*_1_ and *ω*_2_ in the feature map *V*, and ReLU represents Rectified Linear Unit activation function. Equation (5) can realize the information interaction between channels by one-dimensional convolution with convolution kernel size of *T*. The specific relationship is as follows:

(5) $$\begin{array}{c} \omega =\xi \left(C1D_{T}\left(V\right)\right), \end{array}$$

where *C*1*D* represents one-dimensional convolution; there is a mapping *θ* between *T* and *C*, where an exponential function with the base of 2 is used to represent the nonlinear mapping relationship:

(6) $$\begin{array}{c} C=\theta \left(T\right)=2^{\left(\lambda *T-a\right)}, \end{array}$$

where *C* is the channel dimension and *T* is the adaptive kernel size. The relationship size of *T* and *C* is as follows:

(7) $$\begin{array}{c} T=\mu \left(C\right)={\left|\frac{\log_{2}\left(C\right)}{\beta }+\frac{m}{\beta }\right|}_{\text{odd}}, \end{array}$$

where ||_odd_ represents the nearest odd and parameters *β* and *m* are set to 2 and 1. In conclusion, CSAM and PSAM both use average pooling to calculate input features *F*, and the calculation formula of CPASM is as follows:

(8) $$\begin{array}{c} F^{\prime }=\text{CPASM}\left(F\right)=\text{PSAM}\left(F\right)⊗\text{CSAM}\left(\text{PSAM}\left(F\right)\right), \end{array}$$

where ⊗ represents convolution operations, PSAM represents position self-attention mechanism, CSAM represents channel self-attention mechanism, and *F*′ is output feature map.

### 4.3. Construction of the Network Framework

In the first convolution layer, channel self-attention mechanism (CSAM) module is embedded, named first layer. In each dense block of density block, channel self-attention mechanism (CSAM) module is embedded, named DCSAM block layer. Training transition layer is reserved without any modification. After each transition layer, a self-attention mechanism CPSAM module integrating channel self-attention mechanism (CSAM) and position self-attention mechanism (PSAM) is embedded.  Figure 4 describes the network architecture of DCPSNET, and Table 3 shows the relevant parameters of DCPSNET.

### 4.4. Loss Function

There are many loss functions used in convolutional neural network to solve classification problems, such as cross entropy loss function, hinge loss function, ramp loss function, and center loss function. Using different loss functions in different situations can make the model learn more features. If the loss function is small, it indicates that the deep learning model is close to the real distribution of data, and then the model has good performance; if the loss function is large, it indicates that the deep learning model is different from the real distribution of data, and then the performance of the model is poor. In this paper, navel orange pest recognition is a multiclassification problem. In the process of network training, cross entropy is used as the loss function in network training, which is expressed as in the following equation:

(9) $$\begin{array}{c} L\left(n,c\right)=-n\left[c\right]+\log\left(\sum_{k=1}^{c}\exp\left(n\left[k\right]\right)\right). \end{array}$$

Here, *L*(*n*, *c*) is the cross entropy, *c* is the sample label, and *n*[*k*] is the one-bit effective coding representation of the sample label. Considering that the samples are unbalanced and the data sets of individual samples are too few, the accuracy of the model can be effectively improved by setting different types of weight ratio training model. In combination with equation (10), weight is added to simplify the equation:

(10) $$\begin{array}{c} L\left(n,c,\delta \right)=\delta \left[c\right]\left(-n\left(c\right)+\log\sum_{k=1}^{c}\exp\left(n\left[k\right]\right)\right), \end{array}$$

where *δ*[*c*] is the weight vector of the corresponding category. In this paper, according to the imbalance of the pest image, *δ*[*c*]=[0.3, 0.1, 0.1, 0.1, 0.3, 0.3, 0.1].

## 5. Analysis of Experimental Results

### 5.1. Experimental Environment and Model Parameter Setting

In this paper, we use the PyTorch framework to implement the experiment on the operating system Ubuntu 20.04.2 LTS, running memory 31.3Gib, processor AMD @ Ryzen 95900 × 12 core processor × 24, disk capacity 3.0 TB, 1 NVIDIA RTX 3070Ti 8G graphics card, and use CUDA11.2 and cuDNN as support.

At present, there are many ways to train the network model, including randomly initializing the weights of all networks and also using the network weight parameters pretrained on other networks. In addition, in order to further study the performance of the proposed program, this paper selects four influential convolutional neural networks for comparison, namely, AlexNet [26], Vgg19 [27], ResNet-18, and DenseNet-121.

In this paper, we use the Adam optimized cross entropy loss function proposed by Kingma and Ba [28] to train the optimal model. Combining the advantages of AdaGrad and RMSProp, Adam comprehensively considers the first moment estimation (mean value of gradient) and the second moment estimation (variance of gradient) of gradient and calculates the update step. The step size is shown in the following equation:

(11) $$\begin{array}{c} \delta_{i+1}=\frac{\delta_{i}-\eta *\overset{⌢}{m_{i}}}{\sqrt{\overset{⌢}{v_{i+1}}}+\varepsilon }, \end{array}$$

where *δ* is the step, *τ* is the weight, *i* is the class index, *η* is the learning rate, *m* is the first moment estimation of the correction deviation, and *v* is the second moment estimation of the correction deviation.

### 5.2. Evaluating Indicator

The model is evaluated by the commonly used top-1, top-5 accuracy rate, top-1 loss rate, accuracy rate, confusion matrix, kappa coefficient, and other indicators in the image classification task. Top-1 describes the category with the highest probability in the final output probability vector as the prediction category. If the prediction category is consistent with the real category, the prediction is correct; otherwise, the prediction is wrong; top-5 describes the top five categories of the largest probability in the final probability vector, in which the prediction is correct as long as the real category is included. Kappa coefficient is calculated by confusion matrix.

### 5.3. Analysis of Experimental Results

In the training, the batch size of the network is set to 25, the number of iterations is set to 30, and the learning rate is set to 10^−4^. In this paper, four classical CNN models are trained, and a series of experiments are carried out on the data set of this paper. The accuracy of top-1 is shown in Figure 5, and the loss rate of top-1 is shown in Figure 6.

As can be seen from Table 4, after 30-epoch training, the highest top-1 and top-5 rates of DCPSNET, respectively, are 94.275% and 99.997%, and the worst top-1 rate of AlexNet is only 87.536%. In this paper, space complexity is represented by the number of parameters of the model, as shown in Table 4; the number of parameters of DenseNet-121 is the smallest, and that of AlexNet is the largest, and the number of parameters of DCPSNET is 9.995 M, which is more than 3.034 M of DenseNet-121.

After 30 iterations of training, the optimal models of five networks are saved. 227 pictures of diseases and pests of navel orange in the orchard scene were selected as the test set.  Figure 7 clearly shows the accuracy and kappa value of each network in the test set. The precision trend is the same as that in Table 4. The test accuracy of this model is up to **96.90%**, and kappa value is up to **0.962**.

By counting the number of samples of each network in the test set, we analyze the output results in detail. By calculating accuracy, precision, recall, and F1 measure to measure the performance of the network for navel orange pest identification, the definitions are as follows:

(12) $$\begin{array}{c} \text{accuracy}=\frac{\left(\text{TN}+\text{TP}\right)}{\left(\text{TN}+\text{TP}+\text{FN}+\text{FP}\right)}, \end{array}$$

(13) $$\begin{array}{c} \text{recall}=\frac{\text{TP}}{\left(\text{FN}+\text{TP}\right)}, \end{array}$$

(14) $$\begin{array}{c} \text{specificity}=\frac{\text{TN}}{\left(\text{FP}+\text{TN}\right)}, \end{array}$$

(15) $$\begin{array}{c} \text{precision}=\frac{\text{TP}}{\left(\text{FP}+\text{TP}\right)}, \end{array}$$

(16) $$\begin{array}{c} F1-\text{score}=\frac{2\text{TP}}{2\text{TP}+\text{FN}+\text{FP}}. \end{array}$$

In the above formulas, true positive (TP) represents the number of images accurately classified in each type; true negative (TN) represents the number of accurately classified images of all types except related types; false positive (FP) indicates the number of misclassified images in related types; false negative (FN) is the number of misclassified images of all types except related types.

Figure 8 describes the identification results of DCPSNET in the test set by confusion matrix, and Table 5 shows the results determined by the above measurement method. DCPSNET successfully recognized most of the sample images in each category in the orchard scene, and the images of sunguo and health category were correctly recognized with an accuracy of 100%; 89 of 91 ulcer samples were correctly identified, with an accuracy of 97%; only one sample of leaf miner was identified incorrectly, and the accuracy was 98.2%; among 17 samples, 15 were correctly identified, and the accuracy rate was 99.1%; only two of the 13 samples of anthrax were identified incorrectly, with an accuracy of 98.7%.

The classification of models can be achieved by activating the graph (Grad-CAM) [29]. The results provide a good visual basis. Therefore, for further analysis in this paper, we extract part of the test images. The heat of activation in the comparative experiments of various networks is shown in Figure 9. It can be observed that DCPSNET model is more accurate than the other models. It is very important to judge the correct classification of the plant diseases and pests.

## 6. Conclusion

In this paper, a dense network DCPSNET with attention mechanism is proposed to identify navel orange pests. The experimental results show that the DCPSNET model can accurately recognize most of the navel orange diseases samples except a few other samples in the orchard scene. The recognition accuracy of DCPSNET for spot ulcer samples is 0.970, and that for leaf miner and gray mold samples is 0.982 and 0.991, respectively. Through DCPSNET, most of the navel orange plant diseases and pests were accurately identified, and the impressive performance was achieved on the test image. This shows that the proposed DCPSNET model has an important ability in identifying various navel orange pest types and can be transplanted to other fields, including computer-aided detection and online fault assessment.

In contrast, in the case of different diseases on the same plant, there are also individual identification errors. High clutter background and irregular light intensity affect the feature extraction of navel orange lesion image and also lead to individual misclassification. Because the development of artificial intelligence technology makes it possible to automatically identify plant diseases from the original image, it is very important to use digital image to identify and classify various crop diseases to improve the accuracy of disease diagnosis. Deep learning, especially CNN, can identify most of the visual symptoms related to crop diseases efficiently and effectively. Based on the discussion of the efficiency and attention mechanism of DenseNet, this paper proposes a new DCPSNET network architecture. The model has high accuracy and small scale and can be used to identify the pest types of navel orange. The experimental results show that the model has good performance in identifying different diseases of navel orange crops. For the future work, we plan to deploy the model on portable devices to widely monitor and identify navel orange diseases and pests information and apply it to more practical applications.

## Figures and Tables

**Figure 1:** Typical symptoms of navel orange disease. (a) Fruit canker, (b) canker leaf, (c) sunguo, (d) leaf miner, (e) *Botrytis cinerea*, and (f) anthrax.

**Figure 2:** The main structure of DenseNet. (a) Dense block. (b) Transition layer.

**Figure 3:** The main structure of CPSAM.

**Figure 4:** DCPSNET architecture.

**Figure 5:** Comparison curve of top-1 accuracy rate of each model.

**Figure 6:** Comparison curve of top-1 loss rate of each model.

**Figure 7:** Comparison chart of accuracy and kappa value of each model in test set. (a) Test accuracy (%). (b) Kappa.

**Figure 8:** DCPSNET confusion matrix recognition results.

**Figure 9:** Comparison of thermal activation diagrams of various networks.

**Table 1:** The main symptoms of navel orange diseases and pests.

ID	Disease name	The navel orange disease characteristics		
		Shape	Color	Location
1	Sunguo	Cracking deformities of the fruit	Grayish green at first and then yellowish brown	Fruit
2	Canker	Cork-like protuberance	Yellow, grayish brown	Leaf, shoot, fruit, and sepa
3	Leaf miner	The blade curls to the back	—	Young shoots and young leaves
4	*Botrytis cinerea*	Round or irregular	Yellowish brown	Leaf edge and tip
5	Anthrax	The leaves will be watery and soft rot	Light yellowish brown	Petals, tender leaves, young fruits, and branches

**Table 2:** Data before and after enhancement of various types of navel orange units (source: Zhang).

Label	Types	Original data (sheet)	Enhanced data (sheet)
0	Sunguo	74	1332
1	Canker leaf	225	4050
2	Fruit canker	238	4284
3	Leaf miner	283	5094
4	*Botrytis cinerea*	88	1584
5	Anthrax	69	1242
6	Healthy	180	3240
Total	Seven	1157	20826

**Table 3:** Main parameters of DCPSNET.

Layer name	Type	Input shape	Stride	Output size	Maps	Repeated times
Input layer	Input layer	224 × 224 × 3	—	224 × 224	—	1
First layer	Conv2d	224 × 224 × 3	2	112 × 112	64	1
DCSAM block1	SeparableConv2D	112 × 112 × 64	2	56 × 56	160	6
CSAM	Shortcutconnection	56 × 56 × 160	1	56 × 56	160	1
PSAM	Shortcutconnection	56 × 56 × 160	1	56 × 56	160	1
Transform1	Conv2D + Avpooling	56 × 56 × 160	1	56 × 56	80	1
DCSAM block2	SeparableConv2D	56 × 56 × 80	2	28 × 28	272	12
CSAM	Shortcutconnection	28 × 28 × 272	1	28 × 28	272	1
PSAM	Shortcutconnection	28 × 28 × 272	1	28 × 28	272	1
Transform2	Conv2D + Avpooling	28 × 28 × 272	1	28 × 28	136	1
DCSAM block3	SeparableConv2D	28 × 28 × 136	2	14 × 14	520	24
CSAM	Shortcutconnection	14 × 14 × 520	1	14 × 14	520	1
PSAM	Shortcutconnection	14 × 14 × 520	1	14 × 14	520	1
Transform3	Conv2D + Avpooling	14 × 14 × 520	1	14 × 14	260	1
DCSAM block4	SeparableConv2D	14 × 14 × 260	2	7 × 7	516	16
CSAM	Shortcutconnection	7 × 7 × 516	1	7 × 7	516	1
PSAM	Shortcutconnection	7 × 7 × 516	1	7 × 7	516	1
Final_conv	BN + ReLU	7 × 7 × 258	7	1 × 1	7	1
Linear	Classification	1 × 1 × 7	1	7	1	1

**Table 4:** Experimental results of different methods on the data set.

Models	Top-1 accuracy (%)	Top-5 accuracy (%)	Params (M)
AlexNet	87.536	99.396	57.033
VGG19	90.676	99.710	39.599
ResNet18	92.705	99.565	11.180
DenseNet-121	92.729	99.782	6.961
DCPSNET	94.275	99.997	9.995

**Table 5:** DCPSNET identification results metrics.

Class	Types	Test sample	Correct sample	Accuracy	Precision	Recall	Specificity	F1-score
0	Sunguo	14	14	1.0	1.0	1.0	1.0	1.0
1	Canker leaf	44	43	0.987	0.956	0.977	0.989	0.966
2	Fruit canker	47	46	0.991	0.979	0.979	0.994	0.979
3	Leaf miner	56	55	0.982	0.948	0.982	0.982	0.965
4	*Botrytis cinerea*	17	15	0.991	1.0	0.882	1.0	0.938
5	Anthrax	13	11	0.987	0.917	0.846	0.995	0.88
6	Healthy	36	36	1.0	1.0	1.0	1.0	1.0

## Data Availability

The data used to support the findings of this study are available from the corresponding author upon request.
